The article "Design an Effective Blood Distribution Network with Minimal Impacts on the Environment and Blood Supply Assurance" was published in 2022. Journal: J Environ Public Health.

# Design an Effective Blood Distribution Network with Minimal Impacts on the Environment and Blood Supply Assurance

**DOI:** 10.1155/2022/7117151

**Published:** 2022-08-18

**Authors:** Xiaojin Zheng, Shengkun Qin, Yanxia Zhang

**Affiliations:** School of Economics and Management, Tongji University, Shanghai 200092, China

## Abstract

As the world's population grows, resulting in the aggravating trend of aging population, it brings with it an increase in the demand for blood. Nowadays, in most cities, the blood distribution network is based on a single distribution centre pattern, with the blood centre acting as distribution centre for one-to-one distribution. However, despite its convenience, this pattern has a high frequency of delivery, increased risk of blood shortage, and generates high carbon emissions. This paper aims to understand the real-life problems of the current blood distribution network and to design a more rational blood distribution network by taking the characteristics of the blood supply chain into account. Two blood distribution network patterns are considered, the current single distribution centre pattern and the proposed multiple distribution centre pattern. In order to minimise environmental impacts, we introduce open vehicle routing problem for blood delivery routes planning, using mixed integer programming for modelling, to compare the carbon emissions between the two blood distribution network patterns. Numerical experimental results demonstrate that applying the proposed BDN can reduce carbon emissions by an average of 25.84% and up to 29.59%, and the delivery time in emergency situations is significantly reduced by an average of 33.15%. Such studies are essential for both reducing carbon emissions and safeguarding patients' lives.

## 1. Introduction

Blood is a valuable resource, one of the most important but perishable materials in nature. As many operations in hospitals need blood, it is essential in the treatment of patients and is closely associated with human life. Up to now, there is no other product that can completely replace blood and its derivatives. With the reform of the health system and the expansion of hospitals, the amount of clinical blood consumption is increasing year by year. Due to its irreplaceable role in clinical treatment, the provision of blood to the healthcare industry and the public is crucial, and the management of blood and its products is a major issue of concern to humanity [1].

The perishable nature of blood results in a relatively contradictory situation. On the one hand, blood is wasted when it is beyond its expiry date. According to statistics, the annual blood waste rate has reached more than 10% in recent years; on the other hand, during the peak periods of blood consumption in hospitals, blood shortage occurs, resulting in healthcare delays [2]. Thus, the management of blood is different from that of ordinary items, with conflicting objectives leading to more complexities; a trade-off needs to be made between the cost of shortages and expiry of blood products.

Activities in the blood supply chain can be briefly divided into the donation and collection phase, the inventory phase (including testing, preparation, and storage processes), and distribution and clinical use phase [3, 4], as shown in Figure 1. The key to blood supply chain management is to guarantee supply and reduce waste, thereby improving the performance of the supply chain system [5]. The structure of the blood supply chain network has a significant impact on its performance, with an emphasis on the implications for the environment and the security of blood supply.

At present, blood is tested centrally by the blood centre, which is then responsible for distributing blood to hospitals in most cities. Blood has high requirements for storage and transport conditions and is a perishable item, with different shelf lives for different blood products. Blood distribution is a very important issue that evolves with the growth of urban populations in developing countries. An effective blood distribution system is required to get blood to patients in time. Hence, the blood distribution network (BDN) is critical for blood assurance. From the perspective of supply chain network design, this paper addresses the issue of blood resource allocation and dispatching to achieve optimisation of the BDN, thereby achieving a rapid and effective response to blood demand and ensuring timely treatment of patients.

The difficulty of designing blood supply chain networks is routing planning. Delivery routes are closely linked to carbon emissions, with the more distance a blood delivery vehicle travels and the heavier its load, the more carbon emissions it contributes. The transportation routes of blood products consists of two parts, the first is from the blood collection facilities to the blood centre and the second is from the blood centre to the hospitals. The BDN we study is only the second part. As far as we know, fewer studies have been conducted only on blood distribution routing. This problem is similar to the cold chain logistics problem, so we can draw on relevant research methods and experiences. The transportation problem of blood should be considered separately from that of general materials, considering damage and refrigeration impacts during transportation [6]. A mathematical model of cold chain logistics vehicle routing problem is established and an adaptive genetic algorithm is developed to solve the model [7]. There are also many intelligent algorithms for solving cold chain logistics routing problems, such as ant colony algorithm [8], particle swarm algorithm [9], and so on.

The BDN studied in this paper consists of one blood centre and multiple hospitals. Currently, each hospital orders blood directly from the blood centre, which carries out blood distribution and is responsible for satisfying the demand of all hospitals. It is assumed that the blood centre has sufficient capacity and that the hospitals' demand for blood is random and follows a normal distribution with known means and variances. This BDN pattern is well defined on authority and responsibility, is easy to organise and handle, and performs relatively well in practice. However, as the population grows and with the aggravating trend of aging, demand for blood in hospitals continues to increase, and the problems of this pattern are exposed. This one-to-one distribution pattern between the blood centre and hospitals increases the distance travelled by blood delivery vehicles. When the frequency of distribution increases as the demand for blood increases, it generates significant carbon emissions that can be harmful to the environment.

As a scarce and an important healthcare resource, there is still a need for further research on how to implement reasonable dispatch of blood and ensure its supply, which affects both the safety of patients' lives and has a significant impact on the environment. Optimising the BDN structure is an effective way to improve its performance. Nagurney et al. [10] develop a generalised network optimisation model for the blood supply chain. Sahinyazan et al. [11] design a mobile blood collection system, and they propose a mathematical model to determine the tours of the bloodmobiles, as an extension of the selective vehicle routing problem. Kaya and Ozkok [12] design an effective network for a blood distribution system, with the objective of minimising location, inventory, and routing costs. Motivated by these literatures, we try to design the BDN structure to reduce the environmental impact and enhance the ability to safeguard the blood supply of the BDN.

We attempt to apply a new strategy for centralising hospitals' inventory and build a mathematical model for this pattern. Then, we design a more reasonable BDN by combining the characteristics of the blood supply chain to address the practical problems arising from the current BDN pattern. And, we conduct numerical experiments by using realistic data to verify the strategy effectiveness. The results prove that the proposed BDN pattern can reduce carbon emissions by an average of 25.84% and up to 29.59%, preventing further environmental damage. Meanwhile, it can safeguard the supply of blood, with an average reduction of 33.15% of delivery times in emergency situations. The objectives of this research are to (i) highlight the importance of BDN for environmental and blood supply assurance, (ii) describe the need for better management practice, and (iii) develop a better performing solution.

## 2. Implications of BDN and Existing Pattern

### 2.1. Environmental Implications of BDN

Nowadays, all communities are increasingly concerned about environmental issues. Society in general is becoming increasingly aware of and concerned about the environmental impact of human activities and the indiscriminate use of natural resources [13]. There is a growing interest in reducing the environmental impact of various products and services. The BDN's environmental impact is mainly reflected in the transportation process of blood.

The control of environmental impact is a great challenge for modern transport, especially with the current trend of increasing CO_2_ emissions. The environmental impact of transportation is due to the large amount of fuel it uses, as well as the greenhouse effect caused by fuel consumption and pollution. Green transportation has therefore emerged at all levels of supply chain management and are of increasing value to researchers and organisations, due to the fact that current logistics are centered on economic costs without considering the negative impact on the environment and are not sustainable in the long period [14].

The environmental impact of transportation is reflected in the amount of fuel consumed, which depends mainly on distance and load if other factors such as speed and road conditions are held constant [15]. So in this paper the carbon emissions we consider are determined by both the distance travelled and the weight carried. It can be assumed that carbon emissions are proportional to the distance travelled and the weight carried by the vehicle. The BDN model of direct transport between the blood centre and hospitals increases the distance travelled by blood delivery vehicles. If the vehicle routing problem model is used to plan touring blood delivery routes, the distance travelled can be effectively reduced, thereby reducing carbon emissions.

### 2.2. Blood Supply Assurance Implications of BDN

Blood supply chains play an important role in the healthcare systems. Inventory management and distribution of blood are seen as major components of the cost for blood [16]. The BDN configuration will influence hospitals' inventory management strategies, inventory levels, and transport arrangements. The hospitals' blood demands, distance to the blood centre, and the perishable nature of blood are all factors that need to be considered. Life comes first at all times, and there have been real-life incidents where a patient's life was saved because blood was delivered in time at a hospital near the blood centre. Hence, a well-designed BDN is essential for the effective safeguarding of blood supply.

As the demand for blood products in cities grows gradually, the shortage and surplus of blood is becoming more and more serious. Unlike other alternative resources, blood is an exceptional resource with an irreplaceable and important significance. In BDN, both shortage and surplus of the product should be regulated. Blood shortages indicate that demand of blood is not met, which may lead to untimely treatment and even damage to patients' lives. According to the American Red Cross (ARC), approximately 28.9% of hospitals reported the postponement of surgery in the United States for one or more days due to blood shortages in 2007, which approximately affected 412 patients [17]. On the other hand, blood products have a specific expiry date, which can be costly due to the complexity of the handling process.

An acceptable inventory strategy seeks to maximise demand satisfaction and minimise the amount of units that expire. However, the two goals are conflicting because a larger amount of stored product can better meet the changes in demand but would result in an increased storage time for the products, thus increasing losses due to shelf life [18]. Availability of the needed blood products in the right place on time is critical for clinical treatment. Therefore, hospitals must maintain reasonable inventory levels, and the BDN further determines the hospital's ability to respond to requests for blood supplies.

Furthermore, when there is a sudden increased demand for blood and the hospital's existing inventory levels cannot meet the demand, the blood centre is required to arrange emergency blood deliveries. When hospital inventory levels are low and the distance between the hospital and the blood centre is long, this can lead to serious situations that affect treatment and even endanger patients' lives. The frequency and distance of emergency blood deliveries determines the ability to safeguard the blood supply. The BDN needs to be well designed to ensure that not only the usual blood demands are met but also to provide blood supply assurance in emergency situations.

### 2.3. Single Distribution Centre Pattern

The current BDN structure involves two layers, the blood centre and hospitals. The BDN pattern in most cities is that each hospital sends its order request directly to the blood centre, which responds to the request and dispatches a blood delivery vehicle to transport the blood product to the demand point, as shown in Figure 2. The blood centre is the equivalent of a supplier and hospitals are the equivalent of retailers. So, it can be seen that the blood centre is faced with a set of customers with different consumption rates and needs to ensure that shortages and damages are minimised and carbon emissions are reduced.

In this pattern, each hospital needs to manage its blood inventory. The objective of blood inventory management is to minimize inventory costs while safeguarding service levels, rather than minimizing inventory costs. With regard to blood inventory strategies, different scholars have chosen different strategies, such as the (*Q*, *s*) inventory strategy [19]; the (*R*, *S*) inventory strategy [20]; the (*S*^−1^, *S*) inventory strategy [21], which means that as soon as one unit is used, the inventory is immediately replenished to S; and the NIS replenishment strategy [22], i.e., S young units are assumed to enter the system at the beginning of each period. In addition, there are many studies that use a periodic replenishment strategy [23, 24]. Different inventory strategies have corresponding advantages and disadvantages, which need to be combined with the objectives and characteristics of their models to choose the most appropriate strategy; there is no absolute optimal strategy. As for the replenishment lead time, hospitals typically assess their inventory and send requests when the reorder point are reached, with a short delivery time. Therefore, the lead time equal to zero or a fixed nonzero number are reasonable assumptions [25]. In the management practices studied in this paper, we assume that lead time is zero, and hospitals use (*T*, *S*) periodic replenishment strategy, i.e., hospitals replenish their inventory levels to *S* after a certain period *T*.

There is a huge variation in the amount of blood used by different hospitals, and once blood is distributed to hospitals, inventory levels vary greatly from place to place at different times. On the one hand, because shortages could result in loss of life, large hospitals prefer high inventory levels and order far more blood products than they use, even though this results in higher inventory costs and expiry rates of blood products. And, with their long ordering intervals, the inventory levels in hospital blood banks fluctuate very much during the cycle. It is often the case that hospital blood banks have high inventory levels in the early stages, sometimes even having to purchase additional stock resources to satisfy storage needs, and very low inventory levels in the later stages, requiring an increased number of emergency deliveries and waiting times for patients. On the other hand, some other hospitals with low blood consumption only order almost all the blood products they need on a regular or emergency situation, and the blood centre has to apply emergency delivery. These measures are extremely wasteful of storage resources and expensive blood products, as well as adding additional carbon emissions.

The current BDN pattern suffers from shortages and breakdowns, risking patients' lives. Moreover, point-to-point transportation mode and too frequent emergency transportation generate significant carbon emissions. Hence, there is much room for improvement in BDN management practice.

## 3. Innovative Pattern Utilised at BDN

Many scholars have proposed new design solutions for BDN [10–12, 26], and optimisation of the BDN structure can contribute to an effective improvement in its performance. To address problems created by the current BDN pattern, we consider a new configuration strategy in which some hospitals are selected as local blood banks (LBBs) to store blood and are responsible for meeting the demands of other nearby hospitals, as shown in Figure 3. Therefore, in the proposed BDN, inventory is managed in a centralised way, hospitals no longer keep inventory and each LBB is only responsible for the blood demands within the region.

Decisions in the blood supply chain can be classified into strategic-, tactical-, and operational-level decisions [27]. Traditionally, these different dimensions of decisions are considered separately, but this may lead to some problems due to the interactions between different dimensional decisions [12]. This problem consists of three decisions: the location decision, i.e., which hospitals are selected as LBBs and responsible for satisfying the demands of other hospitals allocated to it, the inventory decision, i.e., how to manage inventory for LBBs and hospitals, and the routing decision, i.e., how to arrange distribution routes from the blood centre to LBBs and from LBBs to hospitals.

A focus of the study is to explore the potential value of switching from the current single blood centre managed inventory system to a multi-centre managed inventory system, reallocating resources and responsibilities between the blood centre and LBBs to more effectively safeguard patients' lives. For BDN, inventory centralisation has significant implications. After inventory centralisation, the structure of BDN changes from two layers to three layers, including the blood centre, LBBs, and hospitals. Where the blood centre is equivalent to the supplier, selected LBBs are equivalent to distribution centres, and other hospitals are equivalent to retailers. The inventory strategy is classified into LBBs and hospitals. We assume that hospitals adopt the (*T*, *S*) replenishment strategy, i.e., replenish inventory to S every period *T*, and the LBBs use the (*r*, *Q*) replenishment strategy, i.e., replenish inventory when it falls to *r*, with a replenishment quantity of *Q*. The order cycle *T* for hospitals without inventory is the same as the cycle for hospitals under the current pattern. Although blood demand is stochastic, the demand of LBBs is relatively stable, so the order cycle for LBBs can be simplified to be *t* times of the hospital order cycle; this is realistic with reasonable parameters *r* and *Q*.

Some literature exists on the centralized management of blood inventory. Based on a study of blood banks in the Chicago area, a modified BDN is proposed, where selected hospitals would retain inventory and other hospitals do not hold inventory [28]. Researchers use the median method to select LBBs that retain inventory, and employ the (*r*, *Q*) inventory strategy to construct an academic model, in which there is only direct transportation between nodes and no consideration of vehicle routing problems. What is more, a new BDN structure is proposed where a number of hospitals maintain centralized inventory to meet their and other neighbouring hospitals' demand; the results show that centralization of inventory is a key factor and can improve the sustainability and flexibility of BDN. The numerical experiments find that reducing the number of hospitals holding inventory from 7 to 3 resulted in a 21% and 40% reduction in expiration and shortage in the blood supply chain, respectively [21]. Hence, we can find that centralising inventory helps to free up pressure on resource utilisation and safeguard the blood supply.

In addition to inventory management, we also have to consider the planning of transport routes. After reviewing the relevant literature, direct transport between points increases the distance travelled, and we believe it is necessary to consider the vehicle routing problem in the BDN. The current one-to-one delivery pattern is created on the basis that blood demand is not fixed and each hospital orders at different times depending on their inventory levels. However, centralised inventory management reduces the effects of stochasticity and therefore continuous delivery routes within a region become feasible. Inspired by the idea of resource sharing, many scholars have introduced the open vehicle routing problem model in their research on green logistics [29, 30], where vehicles do not need to return to the start point after completing all tasks. In this paper, two levels of open vehicle routing problem need to be considered, i.e., from the blood centre to LBBs, and from LBBs to hospitals. We develop a mixed integer programming mathematical model to verify that the proposed solution is effective in reducing carbon emissions of BDN.

### 3.1. Distribution Model

Combining the characteristics of the BDN we study, we develop a mathematical model of the open vehicle routing (OVRP) problem for finding delivery routes of blood delivery vehicles. The definition of sets, parameters, and variables used in the model are shown in Table 1. We now present our mixed integer programming model as follows:

(i) The objective function is to minimise carbon emissions generated by blood delivery vehicles. The first term indicates the carbon emissions generated by the routes between the blood centre and LBBs, and the second term is the carbon emissions generated by the routes between each LBB and the hospitals it serves.
  (1) $$\begin{array}{c} \min\sum_{i\in I}\frac{z_{i}d_{oi}qc}{t}+\sum_{i,j\in N}\sum_{v\in V}R_{ijv}d_{ij}u_{j}c. \end{array}$$
The following constraints are satisfied.
(ii) *z*_*i*_ denotes the number of vehicles from o to LBB *i*.
  (2) $$\begin{array}{c} z_{i}\geq \sum_{j\in N}\frac{y_{ij}u_{j}t}{q},\;\forall i\in I. \end{array}$$
(iii) A hospital can be served by just one LBB.
  (3) $$\begin{array}{c} \sum_{i\in I}y_{ij}=1,\;\forall j\in N. \end{array}$$
(iv) At most *b* LBB can be selected.
  (4) $$\begin{array}{c} \sum_{i\in I}x_{i}\leq b. \end{array}$$
(v) If hospital *i* is selected as LBB, it serves itself.
  (5) $$\begin{array}{c} y_{ii}\geq x_{i},\;\forall i\in I. \end{array}$$
(vi) Hospitals can be allocated to a LBB only if the LBB is opened.
  (6) $$\begin{array}{c} y_{ij}\leq x_{i},\;\forall i\in I,\;\forall j\in N. \end{array}$$
(vii) Hospital *i* can be the start node of vehicle *v* only if it is selected as LBB.
  (7) $$\begin{array}{c} s_{iv}\leq x_{i},\;\forall i\in I,\;\forall v\in V. \end{array}$$
(viii) Each route has only one start node and one end node.
  (8) $$\begin{array}{c} \sum_{i\in I}s_{iv}=1,\;\forall v\in V,\\ \sum_{j\in N}h_{jv}=1,\;\forall v\in V. \end{array}$$
(ix) The variable *a*_*iv*_ indicates that hospital *i* is served by vehicle *v*. The relationship between *a*_*iv*_ and the variable *R*_*ijv*_ is shown as constraints (9), (10).
  (9) $$\begin{array}{c} a_{iv}\geq h_{iv},\;\forall i\in N,\;\forall v\in V, \end{array}$$
  (10) $$\begin{array}{c} a_{iv}\geq R_{ijv}+R_{jiv},\;\forall i,j\in N,\forall v\in V. \end{array}$$
(x) One hospital can be involved in only one route.
  (11) $$\begin{array}{c} \sum_{v\in V}\sum_{i\in N}R_{ijv}=1-x_{j},\;\forall j\in N,\\ \sum_{v\in V}a_{iv}=1,\;\forall i\in N. \end{array}$$
(xi) Except for the start node and the end node, if the vehicle passes through one hospital, it must enter and leave from the hospital.
  (12) $$\begin{array}{c} \sum_{j\in N}R_{ijv}-\sum_{j\in N}R_{jiv}=s_{iv}-h_{iv},\forall i\in N,\forall v\in V. \end{array}$$
(xii) The hospital is allocated to the LBB if the route involves this LBB and this hospital.
  (13) $$\begin{array}{c} a_{iv}+a_{jv}-y_{ij}+x_{i}-1\leq 1,\forall i,j\in N,\forall v\in V. \end{array}$$
(xiii) Recursive constraint. If vehicle *v* drives from hospital *i* to hospital *j*, then the value of *f*_*jv*_ is equal to the value of *f*_*iv*_ plus the distance from *i* to *j*.
  (14) $$\begin{array}{c} f_{jv}\geq \sum_{l\in N}\left(f_{lv}+d_{lj}\right)R_{ljv},\forall j\in N,\forall v\in V. \end{array}$$
(xiv) Vehicle capacity constraints.
  (15) $$\begin{array}{c} \sum_{i\in N}a_{iv}u_{i}\leq q,\;\forall v\in V. \end{array}$$
(xv) Enforce the integrality restrictions on the binary variables and enforce the nonnegativity restrictions on the other decision variables.
  (16) $$\begin{array}{c} x_{i},y_{ij},s_{iv},h_{jv},a_{iv},R_{ijv}\in \left\{0,1\right\},\forall i,j\in N,\forall v\in V,\\ f_{jv}\in {\mathbb{Z}}^{+},\forall j\in N,\forall v\in V. \end{array}$$

### 3.2. Numerical Experiments

Before conducting numerical experiments, it is necessary to deal with the nonlinear terms. Linearise the constraint (14) by the following equation, using *L*_*ljv*_ instead of *f*_*lv*_ *R*_*ljv*_.

(17) $$\begin{array}{c} f_{jv}\geq \sum_{l\in N}\left(L_{ljv}+d_{lj}R_{ljv}\right),\forall j\in N,\forall v\in V,\\ L_{ljv}+M\left(1-R_{ljv}\right)\geq f_{lv},\forall l,j\in N,\forall v\in V. \end{array}$$

This paper considers a BDN to create different instances by varying the number of LBBs and available vehicles and its capacity parameters as the case study. In this BDN, there are 1 blood centre and 60 hospitals; we assume that only large general hospitals are candidate locations for the LBB for experimental fluency, 32 hospitals in total can be selected as LBBs. This is because there are many benefits in choosing these hospitals as LBBs, as they have more storage resources and high blood consumption and are generally in more convenient locations.

The experimental data used in this paper are coordinates of the blood centre and hospitals, which are accessible through Gaode Open Platform; in addition, the hospital demands are generated stochastically according to hospital class. Based on the distances from the blood centre to the hospitals, we get the carbon emissions of the current BDN as 7508.86. By using the commercial Off-the-shelf software ILOG CPLEX with a maximum runtime of 3600 s, the proposed model can be solved efficiently. The comparison results between carbon emissions of current and proposed BDN are shown in Table 2, and the column “Reduced (%)” is obtained from the following equation:

(18) $$\begin{array}{c} \text{Reduced}\left(\%\right)=\frac{CE_{\text{current}}-CE_{\text{proposed}}}{CE_{\text{current}}}, \end{array}$$

where *CE*_current_ and *CE*_proposed_ are carbon emissions of the current and proposed BDN, respectively.

As results indicate, significant carbon emission reductions compared to current BDN can be achieved by using the proposed BDN. Sensitivity analysis of the different parameters shows the following conclusions. The number of available vehicles, the number of available LBBs, and the vehicle load capacity are all positively proportional to the carbon emission reduction. Applying the proposed BDN results in carbon emissions being reduced by an average of 25.84% and up to 29.59%.

We then further explore the benefits of the proposed BDN for blood supply assurance in emergency situations. The blood supply assurance is mainly determined by the blood delivery time, which is a function of the distance between the hospital and the blood centre. The configuration and allocation of each hospital and its blood delivery facility under the two BDN patterns are shown in Figures 4 and 5, respectively. From the two figures, it can be seen that the blood centre'ss service areas under the current BDN cover all hospitals, and in the proposed BDN, each selected LBB only needs to provide service within a certain region. The smaller service radius would contribute to reducing the distance travelled by blood delivery vehicles. Using the distance between the blood centre and hospitals, we calculate that the average response delivery time for the current BDN is 44.53 min. The response delivery time results for the proposed BDN are shown in Table 3, with an average response time of 29.77 min, representing an improvement of 33.15% in response capability.

## 4. Conclusion

In this study, we analyse real-world problems arising from the current BDN, and design a new BDN structure in which OVRP is taken into account to minimise environmental impact and improve blood supply assurance capacity. Our focus is to integrate the blood inventory of selected hospitals, in order to help manage blood inventory effectively, reduce shortage and waste of blood products, and ease the pressure on resource allocation. We select some hospitals as LBBs to manage the inventory while other hospitals have no inventory, and then optimise blood delivery routing decisions on this basis. The BDN is converted from a two-level structure to a three-level structure. These measures can safeguard patients' blood supply, improve treatment effectiveness, and reduce life-saving risks to a certain extent.

For the proposed BDN, we develop a mathematical model and convert the nonlinear terms to linear, developing a mixed integer linear programming model. Then, we use the CPLEX commercial solver to solve this model to find the location of a given number of LBBs, the allocation of hospitals to open LBBs, and the distribution routes of blood delivery vehicles. The results of the numerical experiments demonstrate that applying the proposed BDN can effectively reduce carbon emissions by up to 29.59%, and can improve response capacity by an average of 33.15% in emergency blood delivery situations. And parameters such as the number of LBBs, the number of vehicles available, and their capacity all have a relatively significant effect on the results. The next step in the research can be to standardise the scales for carbon emissions, location costs, and blood inventory management indicators to develop integrated models, or consider not just the BDN but also analyse other stages of the blood supply chain such as collection stages in more detail. In addition, real-time dynamic BDN models can also be constructed in order to respond to potential blood supply emergencies in advance, and this is also worth further research.

## Figures and Tables

**Figure 1:** Blood supply chain network.

**Figure 2:** Current blood distribution network.

**Figure 3:** Proposed blood distribution network.

**Figure 4:** Configuration and allocation of current BDN.

**Figure 5:** Configuration and allocation of proposed BDN.

**Table 1:** Notations used in the model.

Sets:	
*N*	Set of hospitals, *n* ∈ *N*;
*I*	Set of hospitals that can be selected as LBB, *i* ∈ *I*, *I*⊆*N*;
*V*	Set of vehicles, *v* ∈ *V*;

Parameters:	
*M*	a large number;
*o*	City blood center;
*b*	Maximum number of LBBs;
*u*_*j*_	Mean daily demand of hospitals *j*;
*t*	Delivery cycle of LBBs;
*d*_*ij*_	Distance between *i* and *j*;
*c*	Carbon emissions per unit distance per unit weight carried generated by blood delivery vehicles;
*q*	Maximum vehicle capacity;

Decision variables:	
*x*_*i*_	Binary variable. If hospital *i* is selected as LBB, it is equal to 1; otherwise equal to 0;
*y*_*ij*_	Binary variable. If hospital *j* is serviced by LBB *i*, it is equal to 1; otherwise equal to 0;
*h*_*jv*_	Binary variable. If hospital *j* is the end node of vehicle *v*, it is equal to 1; otherwise equal to 0;
*s*_*iv*_	Binary variable. If hospital *i* is the start node of vehicle *v*, it is equal to 1; otherwise equal to 0;
*a*_*iv*_	Binary variable. If hospital *i* is visited by vehicle *v*, it is equal to 1; otherwise equal to 0;
*R*_*ijv*_	Binary variable. If vehicle *v* drives from hospital *i* To hospital *j*, it is equal to 1; otherwise equal to 0;
*f*_*jv*_	Distance of the route of vehicle *v* from the start Node to hospital *j*;
*z*_*i*_	Integer variable. Number of vehicles from o to *i*;

**Table 2:** Comparison of carbon emissions between current and proposed BDN.

*n*	*v*	*b*	*q*	Obj	Reduced (%)
60	10	5	500	5733.97	23.64
60	10	5	1000	5287.03	29.59
60	10	2	500	5989.48	20.23
60	10	2	1000	5386.81	28.26
60	5	2	1000	5443.80	27.50
Average					25.84

**Table 3:** Comparison of emergency response time between current and proposed BDN.

*n*	*v*	*b*	*q*	Response time	Reduced (%)
60	10	5	500	34.38	22.79
60	10	5	1000	27.26	38.78
60	10	2	1000	28.34	36.36
60	5	2	1000	31.01	30.36
60	5	5	1000	27.84	37.48
Average				29.77	33.15

## Data Availability

Coordinate data for the blood centre and hospitals are accessible through Gaode Open Platform.

## References

[1] Ahmadimanesh M., Tavakoli A., Pooya A. (2020). Designing an optimal inventory management model for the blood supply chain: synthesis of reusable simulation and neural network. *Medicine*.

[2] Hu B. Y., Chen X. (2011). Study on optimization of blood center inventory system based on simulation technology. *Industrial Engineering & Management*.

[3] Liu L. C. (2017). Research on blood inventory management based on supply chain perspective. *Sci-Tech Innovation and Productivity*.

[4] Piraban A., Guerrero W. J., Labadie N. (2019). Survey on blood supply chain management: models and methods. *Computers & Operations Research*.

[5] Hu B. Y., Chen X. (2016). Optimization of blood supply chain with option contracts under supply and demand uncertainty. *Systems Engineering-Theory & Practice*.

[6] Ma Z. Q., Sun Y. P., Li Z. (2015). Model and algorithm of vehicle delivery of blood in the area. *Logistics Engineering and Management*.

[7] Ma X. G., Liu T. J., Yang P. Z., Jiang R. F. (2016). Vehicle routing optimization model of cold chain logistics based on stochastic demand. *Journal of System Simulation*.

[8] Fang W. T., Ai S. Z., Wang Q., Fan J. B. (2019). Research on cold chain logistics distribution path optimization based on hybrid ant colony algorithm. *Chinese Journal of Management Science*.

[9] Chen J. M., Zhou N., Wang Y. (2018). Optimization of multi-compartment cold chain distribution vehicle routing for fresh agricultural products. *Systems Engineering*.

[10] Nagurney A., Masoumi A. H., Yu M. (2012). Supply chain network operations management of a blood banking system with cost and risk minimization. *Computational Management Science*.

[11] Sahinyazan F. G., Kara B. Y., Taner M. R. (2015). Selective vehicle routing for a mobile blood donation system. *European Journal of Operational Research*.

[12] Kaya O., Ozkok D. (2020). A blood bank network design problem with integrated facility location, inventory and routing decisions. *Networks and Spatial Economics*.

[13] Toro E. M., Franco J. F., Echeverri M. G. (2017). Green open location-routing problem considering economic and environmental costs. *International Journal of Industrial Engineering Computations*.

[14] Lin C., Choy K. L., Ho G. T., Chung S. H., Lam H. Y. (2014). Survey of green vehicle routing problem: past and future trends. *Expert Systems with Applications*.

[15] Xiao Y., Zhao Q., Kaku I., Xu Y. (2012). Development of a fuel consumption optimization model for the capacitated vehicle routing problem. *Computers & Operations Research*.

[16] Aledort L. M., Broder M. S., Busch M. P. (2005). The cost of blood: multidisciplinary consensus conference for a standard methodology”. *Transfusion Medicine Reviews*.

[17] Whitaker B. I., Green J., King M. R. (2007). The 2007 national blood collection and utilizatio survey: report. https://www.researchgate.net/publication/210328395_The_2007_National_Blood_Collection_and_Utilizatio_Survey_Report.

[18] Baesler F., Nemeth M., Martínez C., Bastías A. (2014). Analysis of inventory strategies for blood components in a regional blood center using process simulation. *Blood Management*.

[19] Ma Z. J., Zhou Y. F. (2018). Location-inventory problem for national strategic blood reserves. *Journal of Management Sciences in China*.

[20] Dillon M., Oliveira F., Abbasi B. (2017). A two-stage stochastic programming model for inventory management in the blood supply chain. *International Journal of Production Economics*.

[21] Hosseinifard Z., Abbasi B. (2018). The inventory centralization impacts on sustainability of the blood supply chain. *Computers & Operations Research*.

[22] Civelek I., Karaesmen I., Scheller-Wolf A. (2015). Blood platelet inventory management with protection levels. *European Journal of Operational Research*.

[23] Gunpinar S., Centeno G. (2015). Stochastic integer programming models for reducing wastages and shortages of blood products at hospitals. *Computers & Operations Research*.

[24] Puranam K., Novak D. C., Lucas M. T., Fung M. (2017). Managing blood inventory with multiple independent sources of supply. *European Journal of Operational Research*.

[25] Dehghani M., Abbasi B. (2018). An age-based lateral-transshipment policy for perishable items. *International Journal of Production Economics*.

[26] Liu W. Q., Ke G. Y., Chen J., Zhang L. M. (2020). Scheduling the distribution of blood products: A vendor-managed inventory routing approach. *Transportation Research Part E*.

[27] Osorio A. F., Brailsford S. C., Smith H. K. (2015). A structured review of quantitative models in the blood supply chain: a taxonomic framework for decision-making. *International Journal of Production Research*.

[28] Daskin M. S., Coullard C. R., Shen Z. J. M. (2002). An inventory-location model: formulation, solution algorithm and computational results. *Annals of Operations Research*.

[29] Wang Y., Assogba K., Fan J., Xu M., Liu Y., Wang H. (2019). Multi-depot green vehicle routing problemwith shared transportation resource: integration of time-dependent speed and piecewise penalty cost. *Journal of Cleaner Production*.

[30] Dukkanci O., Kara B. Y., Bektas T. (2019). The green location-routing problem. *Computers & Operations Research*.

